# Therapeutic Effect of Ultrasound-Guided Peripherally Inserted Central Catheter Combined with Predictive Nursing in Patients with Large-Area Severe Burns

**DOI:** 10.1155/2022/1019829

**Published:** 2022-07-31

**Authors:** Baiyan He, Aiqiong Zhang, Shuting He

**Affiliations:** ^1^Department of Burn and Plastic Surgery, Central Hospital of the First People's Hospital, Chenzhou, 423000 Hunan, China; ^2^Intervention Room, South Hospital of the First People's Hospital, Chenzhou, 423000 Hunan, China

## Abstract

This study was aimed to explore the application value of ultrasound-guided peripherally inserted central catheter (PICC) combined with predictive nursing in the treatment of large-area severe burns. 88 patients with large-area severe burns who visited hospital were chosen as the research objects. They were randomly divided into the observation group and the control group, with 44 cases in each. The patients in the observation group were treated with ultrasound-guided PICC combined with predictive nursing, while those in the control group were treated with traditional PICC and nursing methods. Then, the anxiety of patients was compared between groups by the Self-rating Anxiety Scale (SAS), while the depression was compared by the Self-rating Depression Scale (SDS). The pain of the patients was analyzed by the McGill Pain Questionnaire (MPQ), and a self-made nursing satisfaction questionnaire was adopted to evaluate the nursing satisfaction. The surgery-related indicators of the patients were detected and recorded (the success rate of one-time puncture, the success rate of one-time catheter placement, incidence of complications, heart rate, blood pressure, etc.). The success rates of one-time puncture (93% vs. 86%) and of catheter placement (95% vs. 81%) in the observation group were significantly higher than those in the control group, *P* < 0.05. The pain scores of the observation group were much lower than those of the control group at each time period, *P* < 0.05. The number of patients with negative emotions such as anxiety and depression in the observation group was markedly less than that in the control group. The incidence of complications in the observation group was notably lower than that in the control group (4.5% vs 18%), *P* < 0.05. The nursing satisfaction of the observation group was significantly higher than that of the control group (93% vs 79.5%), *P* < 0.05. In conclusion, ultrasound-guided PICC and predictive nursing had high clinical application values in the treatment of patients with large-area severe burns.

## 1. Introduction

Burns bring patients a huge impact on health, life, work, and study. It will weaken the social labor force and increase the economic burden on the family and society. Statistics show that the incidence of burns in China is much higher than that in oversea countries [1]. Generally, burns are classified into four grades: first-degree burns, superficial second-degree burns, deep second-degree burns, and third-degree burns. The specific clinical manifestations of each grade are as follows. For the first-degree burns, the mild burns are generally characterized by mild redness, swelling, and heat pain, with no blisters and no skin damage. It can usually recover to normal within a week without any scarring, but the color of local skin may be darker in a short term. For superficial second-degree burns, blisters of different sizes are formed, and the blister fluid is clear and transparent, which is pale yellow or egg white-like fluid. The ruptured blisters expose a rosy and moist wound [2]. Patients may experience significant pain and local redness and swelling. The wound usually heals in 1-2 weeks without scarring, but sometimes the newly grown skin may have pigment changes. For deep second-degree burns, there is local swelling, and the epithelial tissue turns to be white or brownish-yellow. There are also scattered small blisters; the wound of the ruptured blisters is slightly wet with the color of red and white or red in white. Many red dots or small vascular branches can be observed, the cutaneous sensation is insensitive, and the pain is not obvious. If there is no infection, the healing generally takes about 3-4 weeks. In the event of infection, not only the healing time will be prolonged but also scars will be left after healing. For the third-degree burns, the wound surface is dry and is in waxy white, brown, or charcoal black, with no blisters and no pain. It is tough and leather-like, and thick vascular network coagulates under the eschar, which is caused by venous embolism in the fat layer. In summary, the second- and third-degree burns pose a serious threat to the life and health of patients. In addition, the prognosis of patients is generally very poor, and the treatment time is relatively long. Therefore, the treatment and nursing for burns take a long-term and difficult process [3].

Since burns can cause extensive damage to the protective barrier of the skin, further loss of body fluids can occur. Clinically, long-term fluid supplementation, anti-infection, and postoperative repair are often required for patients. This process typically takes months or even years. Intravenous infusion is commonly used for fluid supplementation in clinical practice. However, the scarred skin formed in burn patients often makes it difficult to find veins, which increases the difficulty of venipuncture. The general puncture requires alternation repeatedly [4]. These can cause great suffering to patients and increase the difficulty of clinical nursing. Therefore, finding a method that can relieve the pain of patients and enable long-term infusion administration is a hot topic of current clinical research [5]. For peripherally inserted central catheter (PICC), the tip of the catheter is located in the superior vena cava, which can quickly dilute the drug. Thus, it can avoid problems such as phlebitis and drug leakage caused by tissue necrosis [6, 7]. In addition, PICC also has the advantages of long indwelling time as well as no risk of pneumothorax and arterial injury [8, 9]. With the development of imaging technologies such as ultrasound, the improved Seldinger PICC placement technique under ultrasound guidance has been gradually derived [10]. A large number of clinical studies have shown that the success rate of traditional PICC placement is only 78%, the success rate of PICC placement using optimized Seldinger technique alone is 84%, and that of optimized ultrasound-guided Seldinger PICC placement reaches 98%. In general, ultrasound-guided optimized Seldinger technique for PICC placement has the wide and good clinical applications. However, there is no direct report worldwide about its application in patients with large-area severe burns [11]. Therefore, further in-depth research is needed on its application effect in patients with large-area severe burns.

There are also some defects and deficiencies in the optimized Seldinger PICC placement technique guided by ultrasound. For example, venipuncture and blade dilation are required during catheter placement, which can cause local tissue damage and pain in patients [12]. Pain caused by ultrasound-guided optimized Seldinger PICC placement can lead to a series of physiological and pathological changes, and these changes are important factors causing postoperative complications. Therefore, it is necessary and urgent to take appropriate nursing intervention methods to improve the quality of life and prognosis of severely burned patients. Predictive nursing is a method that is widely used worldwide and has been recognized and confirmed by many scholars [13]. Predictive nursing, conducted by some foreign scholars, has reduced the incidence of coronary heart disease by 50%. For patients with advanced head and neck tumors, some scholars have adopted predictive enteral nutrition support nursing, and found that this nursing measure can make the patients with neck tumors nourished. Researches by domestic scholars show that predictive nursing can improve the comfort, satisfaction, and compliance of clinical treatment. There are many similar studies [14]. From the above, predictive nursing has achieved good outcomes in clinical work and has been widely promoted. It can effectively relieve the negative moods of patients and reduce the incidence of complications. However, all the existing related researches in the world directly reported the application of predictive nursing in the PICC of burn patients under the ultrasound-guided modified Seldinger technique. As for the application effect of the modified Seldinger technique in the PICC of burn patients under the guidance of ultrasound, further research is needed [15].

The patients with large-area severe burns were preselected as the research objects in this research, so as to explore the application value of ultrasound-guided PICC placement combined with predictive nursing in the treatment. It was expected to provide reference and basis for the clinical treatment of related diseases as well as the application of related technologies.

## 2. Research Methods

### 2.1. Objects

In this study, 100 patients with severe burn admitted to the hospital from July 2020 to January 2022 were selected and randomly divided into control group and observation group, with 50 cases in each. The ultrasound-guided PICC combined with predictive nursing was given in the observation group, while the control group received traditional PICC combined with nursing. Inclusion criteria required the patients had an age of 18-66 years old, no skin damage to the auricle, no history of alcohol allergy, and PICC placement for the first time. Besides, the patients were suitable for the indications of PICC; they had no mental illness and could correctly express pain. No systemic or local pain relief measure was taken for 24 hours before PICC placement. Exclusion criteria were as follows. The patients received deep venous catheter placement (intravenous access port, subclavian or internal jugular, and femoral venous catheter placement). The diameter of the basilic vein, brachial vein, and median cubital vein under B-mode ultrasound was <5 mm^2^. The patients suffered from upper extremity hemiplegia, had a history of surgery, or had an unsuccessful one-time venipuncture. They received radiotherapy, chemotherapy, drugs, surgery, or other treatments that could relieve pain during the research. The informed consent forms were obtained from patients, and this study had been approved by ethics committee of hospital.

### 2.2. PICC Puncture Methods

In the control group, ordinary deep vein puncture was adopted for PICC placement. A disposable puncture catheter was used, the patient was in a supine position, the arm to be catheterized was abducted by 90°, and the vein below the elbow was selected for puncture. After the blood vessel is selected, sterilization and draping were carried out. Puncture was performed with a puncture needle, the needle core was withdrawn after the venous return was observed, and the catheter was sent into along the outer cannula of the puncture needle until to the predetermined length. Then, the guide wire was withdrawn, the catheter was connected to the installer, and the sterile saline gauze was used to clean the skin around the puncture point. The puncture point was covered with sterile gauze and fixed with transparent application. After the catheter was fixed, it was positioned under X-ray.

In the observation group, the patients underwent PICC placement using the ultrasound-guided technique. The body position and disinfection method were the same as those in the control group. The vein below the elbow was selected for puncture. The approximate position of the vein was displayed on the transverse section under color Doppler ultrasonic apparatus. Then, the longitudinal section was scanned to observe the blood flow, wall thickness, and blood vessel diameter of the vein. It was turned to the transverse section, the midpoint of the probe was located at the same point as the transverse section of the vein, and this point was marked, which was just the position on the body surface of the vein. This point was as the starting point, and a point was located after detection every 1 cm. A total of 3 points were located, and the 3 points were kept on the same straight line. After routine disinfection and draping, the lowest located point was the needle insertion point of puncture. The probe was at right angles to the vein as well as to the skin. Under the guidance of ultrasound, the puncture needle and the vein were advanced in parallel. After good blood return was obtained, the position of the needle core was kept unchanged, and the guide wire was put into for 10 cm. After, the puncture angle was reduced, and it was continued to insert the guide wire. The needle core was then withdrawn, the catheter sheath was advanced, and the catheter was placed well.

### 2.3. Nursing Intervention

The patients in the control group received routine nursing. The nursing mainly included admission introduction, medication guidance, routine observation, auxiliary treatment, health education, and other basic nursing care.

The patients in the observation group were given with predictive nursing. A predictive nursing intervention team was established. The team organized team members for nursing knowledge training every week and conducted regular assessments. The specific interventions were as follows. (1) On the basis of fully understanding of the patients' acquisition of knowledge, a systematic knowledge theory system was constructed. Through repeated communications, distribution of brochures, and other methods, the correct cognition of disease understanding in patients was deepened and strengthened. The patients were also helped to establish correct beliefs and attitudes. (2) During the treatment and nursing period, the Self-rating Anxiety Scale (SAS) and the Self-rating Depression Scale (SDS) were adopted for observing and evaluating whether the negative situation occurred in patients. If the patient had depression, anxiety, etc., it was necessary to give a targeted psychological intervention measure, and the intervention was carried out every 7 days for 25 minutes each time. (3) Patients with severe burns might need to stay in bed for a long time, and some negative emotions could also affect the vagus nerve, resulting in constipation. Nursing intervention team needed to carry out reasonable dietary intervention for patients. (4) For nursing after catheter placement, chitin-type wound dressings should be used for fixation, to promote hemostasis and healing at the puncture point as soon as possible. Relevant information was recorded in detail on the catheter maintenance record sheet, including catheter model, batch number, the position of catheter placement, catheter placement length, and other information. The precautions, possible adverse reactions, daily life precautions, and common sense of self-maintenance after catheter placement were explained in detail to the patients and their families. The importance of regularly maintaining the catheter and keeping the catheter in good condition was also expounded.

### 2.4. Observation Indicators

*Pain score*: The McGill pain questionnaire (MPQ) was used for estimation. With standards of the pain rating index (PRI) score (0-3 points), 0 point stood for no pain, 1 point for mild pain, 2 points for moderate pain, and 3 points for severe pain. Under the Present Pain Intensity (PPI) scoring (0-5 points), no pain, mild pain, pain causing discomfort, moderate pain, severe pain, and unbearable pain were indicated by 0, 1, 2, 3, 4, and 5 points, respectively. The observation and comparison were at six time points, including local anesthesia, venipuncture, withdrawal of puncture needle, blade expansion, vascular sheath insertion, and vascular sheath withdrawal.

*Anxiety situation*: The SAS was adopted for the evaluation of patients' anxiety, with a score of 0 to 100. The SAS standard score <50 indicated no anxiety, 50-59 indicated mild anxiety, 60-69 meant moderate anxiety, and 70 and above represented severe anxiety. The comparison was made before nursing and 15 days after nursing intervention, respectively.

*Depression*: As SDS was used for evaluation, SDS standard score <53 meant no depression. 53-62, 63-72, and ≥73 were denoted as mild depression, moderate depression, and severe depression, respectively. It was compared before nursing as well as 15 days after nursing intervention.

*Surgery-related indicators*: The success rate of one-time puncture, the success rate of one-time catheter placement, the incidence of complications, and the basic physiological indicators such as heart rate (measured by the doctors using a stethoscope) and blood pressure (measured with a sphygmomanometer) of the patients in the two groups were recorded. These were compared 15 days after nursing intervention.

*Bacterial culture*: The condition of bacterial infection was compared between the two groups during the nursing intervention period.

### 2.5. Statistical Methods

The observed data were filled in the observation table, and the values were entered into the SPSS11.0 software for statistical analysis. The data were statistically described by the mean ± standard deviation, and the measurement data were analyzed by *t* test. The scores before and after nursing intervention were compared using paired-sample *T* test within the same group, while the scores were compared using the independent-sample *T* test between the groups. *P* < 0.05 meant a difference was statistically significant.

## 3. Results

### 3.1. General Information

The general data of the two groups of patients are listed in Table 1. The observation group included 28 male patients and 22 female patients, with an average age of 44.2 ± 9.8 years old. In the control group, 30 male patients and 20 female patients were included, having an average age of 55.3 ± 11.3 years old. There was no statistical difference in these general data between two groups, *P* < 0.05.

### 3.2. Comparison of the Success Rates of Puncture and Catheter Placement

The success rates of puncture and catheter placement were compared between the two groups as shown in Figure 1. The number of successful one-time puncture was 48 (96%) and 41 (82%), respectively, in the two groups. The success rate of one-time catheter placement was 47 (94%) and 39 (78%), respectively. The success rates of both one-time puncture and one-time catheter placement were markedly higher in the observation group than those in the control group, *P* < 0.05.

### 3.3. Comparison of Pain Scores

The comparison results of the MPQ pain scores in the two groups are displayed in Figure 2. The MPQ scores of the two groups of patients were 36.3 ± 9.88 and 35.5 ± 11.3, respectively, before nursing intervention, with no significant difference, *P* > 0.05. The MPQ scores after nursing intervention turned to be 18.6 ± 7.11 and 28.9 ± 6.3, respectively. After intervention, the MPQ score of the observation group was greatly lower than that of the control group, *P* < 0.05.

### 3.4. Comparison of Anxiety and Depression

The anxiety condition of the two groups of patients is presented in Figure 3. Before intervention, the number of patients without anxiety, mild anxiety, moderate anxiety, and severe anxiety were counted as 6, 24, 18, and 2, respectively, in the observation group. Those were 7, 23, 19, and 1, respectively, in the control group. The SAS scores of the two groups were 55.3 ± 11.3 and 56.1 ± 9.6, respectively, having no statistical difference in anxiety between the two groups, *P* > 0.05. After nursing intervention, there were 18, 30, 2, and 0 patients with no anxiety, mild anxiety, moderate anxiety, and severe anxiety, respectively, in the observation group, while 13, 16, 19, and 2 patients in control group, respectively. The SAS scores of the two groups became 40.3 ± 8.7 and 55.1 ± 10.2, respectively. The anxiety of patients in the observation group was pretty milder than that of the control group, *P* < 0.05.

The comparative results of depression of patients in the two groups are displayed in Figure 4. The number of patients with no, mild, moderate, and severe depression was counted to be 11, 30, 5, and 4, respectively, before intervention in the observation group. 13, 28, 6, and 3 patients got no, mild, moderate, and severe depression, respectively, in the control group. The SDS scores of the two groups were 60.2 ± 9.9 and 62.2 ± 10.2, respectively, before intervention, without a statistical difference in anxiety between the two groups as *P* > 0.05. After nursing intervention, 25, 20, 4, and 1 patient in the observation group and 8, 10, 30, and 2 patients in the control group had no depression, mild depression, moderate depression, and severe depression, respectively. The SDS score was 48.8 ± 9.9 in the observation group while 60.2 ± 11.2 in the control group. The depression status of patients in the observation group was remarkably milder than that in the control group, *P* < 0.05.

### 3.5. Comparison of Physiological Indicators

The physiological indicators of patients in the two groups are compared in Figure 5. The systolic blood pressure before nursing intervention was 115 ± 11.3 mmHg in the observation group and 116 ± 10.2 mmHg in the control group, showing no significant difference between the groups. After intervention, the systolic blood pressure turned to be 110 ± 8.8 mmHg and 125 ± 9.3 mmHg, respectively, in the observation and control groups. The diastolic blood pressure before intervention was 68.8 ± 5.2 mmHg and 69.3 ± 6.7 mmHg, respectively; not a significant difference was found between the groups. The diastolic blood pressure after intervention was 69.3 ± 10.2 mmHg and 73.8 ± 11.4 mmHg in the observation and control groups, respectively; a significant difference was shown between groups, *P* < 0.05. The heart rates were 70.3 ± 4.4 beats/min and 70.8 ± 5.2 beats/min before intervention in the two groups, suggesting no significant difference between groups. The heart rates after intervention were 70.8 ± 3.8 beats/min and 79.3 ± 3.7 beats/min, respectively, in the observation and the control groups, with a significant difference between groups for *P* < 0.05.

### 3.6. Comparison of Complications

The incidence of complications in the two groups is shown in Figure 6. There were 0, 1, 1, and 0 patients with local hematoma, local infection, thrombosis, and phlebitis, respectively, in the observation group. The incidence of complications was counted to be 4.5% in the observation group. 2, 3, 2, and 1 patient got the complications, respectively, in the control group; thereout, the incidence of complications was 18%.

### 3.7. Comparison of Nursing Satisfaction

The comparative results of nursing satisfaction in the two groups are presented in Figure 7. There were 36, 11, and 3 patients satisfied, basically satisfied, and dissatisfied, respectively, in the observation group. The satisfied rate reached 94%. In the control group, 24, 17, and 9 patients were satisfied, basically satisfied, and dissatisfied, respectively, with the satisfied rate of 82%. The satisfaction of the observation group was observably higher than that of the control group, *P* < 0.05.

### 3.8. Comparison of the Incidence of Bacterial Infection

The incidence of bacterial infection was compared between the two groups. 3 (6%) patients got bacterial infection in the observation group, while bacterial infection occurred in 9 (18%) patients in the control group. The number of patients with bacterial infection in the observation group was considerably less than that in the control group, *P* < 0.05.

## 4. Discussion

Not only affect burns life and health but even destroy the patients' life, work, and study. Burns will weaken the social labor force and also lay an increased economic burden on the family and the society [16, 17]. The protective barrier of large areas of the skin is damaged when a burn occurs, which can lead to a massive loss of body fluids. Thus, long-term fluid supplementation, anti-infection, and postoperative repair are often required for patients in clinical practice. Typically, this course takes months or even years. These procedures are generally completed by intravenous infusion. However, burn patients generally have scarred skin, which makes the veins difficult to find, greatly increasing the difficulty of venipuncture. In addition, conventional puncture or central venous catheter requires repeated alternation and replacement in a short time period [18]. These problems and shortcomings often bring pain to patients and increase the difficulty of clinical nursing. On the basis of the treatment characteristics of burns, it is indispensable and urgent to find a method that can relieve the pain of patients, avoid local skin infection, and achieve good long-term infusion administration as well [19].

PICC refers to the technique of inserting a central venous catheter through peripheral vein puncture, so that the tip of the catheter reaches the superior vena cava or subclavian vein [20–22]. As the tip of PICC is in the superior vena cava, the drugs can be quickly diluted, thus avoiding tissue necrosis caused by phlebitis and drug leakage [23, 24]. Moreover, PICC placement is generally operated independently by a professional nurse, having the advantages of long indwelling time and no risk of pneumothorax as well as arterial injury. With the development of imaging technologies including ultrasound, the optimized Seldinger PICC placement technique has been derived gradually under ultrasound guidance [25]. In a large number of clinical studies, the success rate of traditional PICC placement is only 78%, that rises to 84% as modified Seldinger technique was used, and reaches 98% using optimized ultrasound-guided Seldinger PICC placement [26, 27]. The ultrasound-guided optimized Seldinger technique has a wide range of great clinical applications for PICC placement. Thereout, PICC placement has a high application value in burn treatment. Therefore, in this work, patients with severe burns were selected as the research objects, and were randomly divided into the observation group and the control group. In the observation group, ultrasound-guided PICC technology was utilized for catheter placement, while traditional PICC was adopted in the control group. The success rate of one-time puncture (93% vs. 86%) and the success rate of one-time catheter placement (95% vs. 81%) in the observation group were notably higher than those in the control group, *P* < 0.05. It suggested that the application value of ultrasound-guided PICC technology was much higher than that of traditional catheter placement technology in the treatment of severe burns. This was consistent with the findings of previous related studies.

In spite of many advantages of the ultrasound-guided optimized Seldinger technique for PICC placement, it also has some flaws and deficiencies. Venipuncture, blade dilation, etc. are needed during catheter placement, and these PICC operations can cause local tissue damage as well as pain to the patients [28]. With the continuous development of pain specialty, pain has become the fifth vital sign after the four vital signs of breathing, pulse, blood pressure, and body temperature [29]. Pain caused by PICC placement can bring about a series of physiological and pathological changes, which are important factors for postoperative complications. Therefore, taking appropriate nursing intervention methods is necessary and urgent for severely burned patients, to promote their quality of life and prognosis. Predictive nursing is widely applied and has been recognized by numerous scholars across the world [30]. In this work, patients with large-area severe burns were included as the research objects. The patients were randomly divided into the observation group and the control group. The observation group received ultrasound-guided PICC technology combined with predictive nursing, while traditional PICC combined with traditional nursing was adopted in the control group. The MPQ scores of the observation group were significantly lower than those of the control group at each time period, *P* < 0.05. The patients in the observation group had significantly fewer negative emotions such as anxiety and depression than the control group. The incidence of complications in the observation group was significantly lower than that in the control group (4.5% vs 18%), *P* < 0.05. The nursing satisfaction in the observation group was greatly higher than that of the control group (93% vs 79.5%), *P* < 0.05. In summary, ultrasound-guided PICC and predictive nursing had high clinical application value in the treatment of patients with large-area severe burns. This was consistent with the predictions.

## 5. Conclusion

The patients with severe burns were selected as the research objects and were randomly divided into the observation and the control groups. In the observation group, patients received ultrasound-guided PICC with predictive nursing, while traditional PICC and traditional nursing were given to the control group. The ultrasound-guided PICC and predictive nursing showed high clinical application values in treating large-area severe burns; thus, this work provided a reference and basis for the clinical treatment. However, due to the limited samples and text space, this work still had certain defects. In the future, the samples would be expanded for further research.

## Figures and Tables

**Figure 1:** Comparison of the success rates of puncture and catheter placement in two groups. ^∗^Compared with control group, *P* < 0.05.

**Figure 2:** Comparison of MPQ pain scores of patients between the two groups. ^∗^Compared with control group, *P* < 0.05.

**Figure 3:** Comparison results of anxiety of patients between two groups. (a), (b), and (c) represented before intervention, after intervention, and SAS score, respectively. ^∗^Compared with control group, *P* < 0.05.

**Figure 4:** Comparison results of depression status of patients in two groups. (a) Before intervention. (b) After intervention. (c) SDS score. ^∗^Compared with control group, *P* < 0.05.

**Figure 5:** Comparison of physiological indicators between two groups. (a), (b), and (c) represented systolic blood pressure, diastolic blood pressure, and heart rate, respectively. ^∗^Compared with control group, *P* < 0.05.

**Figure 6:** Comparison of the incidence of complications in two groups. ^∗^Compared with control group, *P* < 0.05.

**Figure 7:** Comparison of nursing satisfaction of patients in two groups.

**Table 1:** General information of patients in the two groups.

Items	Observation group (*n* =50 cases)	Control group (*n* =50 cases)	*X* ^2^/*t* value	*P*
Gender			0.388	0.614
Male	28	30		
Female	22	20		
Age (years old)			0.120	0.133
	44.2 ± 9.8	55.3 ± 11.3		
Nationality			2.131	1.810
Han Chinese	36	38		
Minorities	14	12		
Education level			0.335	0.198
Primary school and below	8	9		
Junior high school	13	11		
High school or technical secondary school	20	21		
College and above	9	9		
Marital status			0.512	0.837
Married	23	25		
Single	17	16		
Divorced	5	4		
Widowed	5	5		
Monthly income per capita (yuan)			0.383	0.193
<1,000	11	10		
1,000-3,000	18	16		
3,001-5,000	16	17		
>5,000	5	7		
Payment method			0.449	0.527
Urban medical insurance	20	21		
Rural cooperative medical care	22	18		
Commercial insurance	5	6		
Self-paying	3	5		

## Data Availability

The data used to support the findings of this study are available from the corresponding author upon request.
